# Evolutionary biology of antimalarial drug resistance: Understanding of the evolutionary dynamics

**DOI:** 10.1097/MD.0000000000041878

**Published:** 2025-03-14

**Authors:** Matthew Chibunna Igwe, Ogbonna Alphonsus Ogbuabor, Emmanuel Ifeanyi Obeagu

**Affiliations:** a Department of Public Health, School of Allied Health Sciences, Kampala International University, Kansanga, Uganda; b Department of Medical Laboratory Science, Faculty of Basic Medical Sciences, College Medicine, Enugu State University of Science and Technology, Enugu, Nigeria; c Department of Medical Laboratory Science, School of Allied Health Sciences, Kampala International University, Kansanga, Uganda.

**Keywords:** antimalarial, biology, drug, evolutionary, resistance

## Abstract

Anti-malarial drug resistance poses a significant challenge to global malaria control efforts, necessitating a deeper understanding of the evolutionary dynamics underlying the emergence and spread of resistance. This study explores how evolutionary theory provides a framework for elucidating the molecular mechanisms and genetic variation within parasite populations that drive resistance evolution. Drawing on recent research findings, we discuss the role of natural selection, genetic diversity, and fitness costs in shaping resistance phenotypes. Additionally, we highlight the implications of evolutionary insights for antimalarial drug policy, treatment guidelines, and future research directions. By integrating evolutionary biology principles with molecular epidemiology, this review aims to inform strategies for combating antimalarial drug resistance and advancing malaria treatment efforts. Using evolutionary theory to understand the dynamics of antimalarial drug resistance at the molecular level, we explored the influence of genetic variation within parasite populations on the emergence and spread of resistance. Antimalarial drug resistance poses a formidable challenge to global malaria control. By applying evolutionary theory to understand the dynamics of resistance emergence and spread at the molecular level, researchers can develop more effective strategies for surveillance, prevention, and treatment of drug-resistant malaria.

## 1. Introduction

Malaria remains a significant global health challenge, with approximately 229 million cases and 409,000 deaths reported in 2019 alone.^[1]^ One of the cornerstones of malaria control is the use of antimalarial drugs, which play a crucial role in reducing the burden of the disease. However, the emergence and spread of antimalarial drug resistance poses a serious threat to these control efforts.^[2]^ Antimalarial drug resistance occurs when Plasmodium parasites, the causative agents of malaria, evolve mechanisms to evade the effects of drugs, rendering them ineffective in treating the disease.^[3]^ This phenomenon has been observed with multiple classes of antimalarial drugs, including chloroquine, sulfadoxine-pyrimethamine, and more recently, artemisinin-based combination therapies (ACTs).^[4,5]^

The emergence of drug-resistant strains compromises treatment efficacy, leading to prolonged illness, increased mortality, and higher healthcare costs.^[6]^ Moreover, drug resistance can undermine malaria control and elimination efforts, as it may lead to the resurgence of transmission and the spread of resistant parasites to new geographic areas.^[7]^ Understanding the evolutionary dynamics of antimalarial drug resistance at the molecular level is essential for devising effective strategies to combat this phenomenon. Evolutionary theory provides a framework for comprehending how genetic variation within parasite populations influences the emergence and spread of drug resistance.^[8]^ The genetic diversity of Plasmodium populations plays a central role in the emergence of drug resistance. High levels of genetic variation, coupled with the parasite’s rapid reproduction rate, facilitate the generation of mutant strains with reduced susceptibility to antimalarial drugs.^[9]^ These mutants can arise through spontaneous mutations in genes encoding drug targets or enzymes involved in drug metabolism.^[10]^

The molecular mechanisms underlying antimalarial drug resistance vary depending on the drug class. For instance, resistance to chloroquine is primarily mediated by mutations in the Plasmodium falciparum chloroquine resistance transporter (pfcrt) gene, which encodes a transporter protein involved in drug accumulation within the parasite’s digestive vacuole.^[11]^ Similarly, resistance to artemisinin and its derivatives has been linked to mutations in the kelch13 (k13) gene, which is associated with decreased drug susceptibility and delayed parasite clearance.^[12]^ Once resistance-conferring mutations emerge within parasite populations, their spread is influenced by several factors, including drug selection pressure, population genetics, and transmission dynamics.^[13]^ Selective sweeps driven by drug usage can lead to the rapid dissemination of resistant genotypes, particularly in areas with high malaria transmission intensity.^[14]^ Additionally, genetic recombination and gene flow between parasite populations contribute to the spread of resistance alleles across geographic regions.^[15]^

## 2. Evolutionary biology in the context of antimalarial drug resistance

Evolutionary biology provides a comprehensive framework for understanding the dynamics of antimalarial drug resistance at the molecular level.^[8]^ This framework incorporates principles of population genetics, natural selection, and genetic variation to elucidate how Plasmodium parasites adapt to selective pressures imposed by antimalarial medications.^[16]^ Population genetics principles are fundamental to understanding the genetic diversity within Plasmodium populations and the emergence of drug-resistant strains.^[17]^ High levels of genetic variation within parasite populations provide the raw material for the evolution of drug resistance mutations.^[18]^ Genetic diversity arises through mechanisms such as mutation, recombination, and gene flow, allowing parasites to explore a vast genetic landscape and adapt to changing environmental conditions, including drug exposure.^[19]^

Natural selection acts on the genetic variation present in Plasmodium populations, favoring the survival and proliferation of parasites with advantageous traits, such as drug resistance mutations.^[20]^ In the presence of antimalarial drugs, parasites carrying resistance-conferring mutations have a selective advantage, as they can survive and replicate despite drug pressure.^[16]^ Over time, these resistant parasites may come to dominate the parasite population, leading to the spread of drug resistance.^[9]^

At the molecular level, drug resistance mutations often involve changes in the genetic sequences encoding drug targets or enzymes involved in drug metabolism.^[21]^ For example, mutations in genes encoding the pfcrt and multidrug resistance protein 1 (pfmdr1) have been associated with chloroquine resistance, while k13 gene have been linked to artemisinin resistance.^[11,12]^

### 2.1. Principles of evolutionary theory in the study of drug resistance

Evolutionary theory provides fundamental principles that underpin the study of antimalarial drug resistance, shedding light on how Plasmodium parasites adapt to selective pressures imposed by drugs. Several key principles, including natural selection, genetic variation, and adaptation, are central to understanding the dynamics of drug resistance emergence and spread.^[8]^

#### 2.1.1. Natural selection

Natural selection acts on the heritable variation present within populations, favoring individuals with traits that confer a fitness advantage in their environment.^[22]^ In the context of antimalarial drug resistance, parasites carrying genetic mutations that confer resistance to drugs have a selective advantage, as they are more likely to survive and reproduce in the presence of drug pressure.^[4]^ Over time, natural selection leads to the enrichment of drug-resistant parasites within the population, driving the spread of resistance.^[20]^

#### 2.1.2. Genetic variation

Genetic variation is the raw material upon which natural selection acts, providing the diversity necessary for populations to adapt to changing environments.^[17]^ Within Plasmodium populations, genetic variation arises through mechanisms such as mutation, recombination, and gene flow.^[18]^ This genetic diversity allows parasites to explore a vast genetic landscape and adapt to selective pressures, including exposure to antimalarial drugs.^[16]^ Understanding the distribution and dynamics of genetic variation within parasite populations is crucial for predicting and managing the emergence of drug resistance.^[23]^

#### 2.1.3. Adaptation

Adaptation refers to the process by which organisms evolve traits that enhance their fitness in a specific environment.^[24]^ In the case of antimalarial drug resistance, parasites adapt to the presence of drugs by acquiring mutations that confer resistance to drug action.^[25]^ These adaptive changes may involve alterations in drug targets, metabolic pathways, or transport mechanisms, allowing parasites to survive and proliferate in the presence of drug pressure.^[26]^ Adaptation to drug pressure is a dynamic process shaped by ongoing interactions between parasites, drugs, and the host environment.^[13]^

### 2.2. Selective pressure of antimalarial drugs on parasite populations

Antimalarial drugs exert selective pressure on Plasmodium parasite populations, driving the emergence of resistant strains through a process governed by evolutionary principles. This phenomenon occurs due to the differential survival and reproduction of parasites with advantageous traits in the presence of drug treatment.^[27]^

#### 2.2.1. Mechanisms of selective pressure

Antimalarial drugs create a selective environment where parasites with genetic mutations that confer resistance to drug action have a survival advantage over susceptible parasites.^[6]^ Mutations in genes encoding drug targets, such as the pfcrt or dihydrofolate reductase, can reduce the binding affinity of drugs, rendering them ineffective against resistant parasites.^[11]^ Parasites may develop mechanisms to bypass or enhance drug metabolism, reducing the concentration of active drug compounds within the parasite and limiting their effectiveness.^[28]^

#### 2.2.2. Dynamics of resistance emergence

Spontaneous mutations occur within parasite populations, leading to the generation of genetic variants with altered drug susceptibility. Under drug pressure, parasites carrying resistance-conferring mutations are selectively favored, allowing them to proliferate and dominate the population.^[4]^ The use of drug regimens in rotational or sequential cycles can inadvertently promote the emergence of drug resistance by exerting fluctuating selective pressures on parasite populations. This cycling can select for preexisting resistant strains or facilitate the evolution of new resistance mutations.^[29]^

#### 2.2.3. Fitness costs of drug resistance mutations (mechanisms of fitness costs)

Drug resistance mutations in Plasmodium parasites can incur fitness costs, which are adverse effects on the parasite’s ability to survive and reproduce in the absence of drug pressure. These fitness costs can influence the spread and persistence of resistance within parasite populations.^[30–32]^ Drug resistance mutations may impair the parasite’s reproductive capacity, leading to decreased rates of replication and transmission. For example, mutations that confer resistance to antimalarial drugs may disrupt essential biological processes, such as DNA replication or protein synthesis, resulting in slower growth rates or lower parasite densities.^[27]^ Drug-resistant parasites may exhibit reduced fitness when infecting hosts who have not been exposed to drug treatment. This phenomenon can arise due to the specific genetic changes associated with drug resistance, which may compromise the parasite’s ability to compete with wild-type parasites in untreated individuals.^[31–33]^ Drug resistance mutations may alter metabolic pathways or cellular functions, leading to trade-offs in parasite fitness. For example, mutations that confer resistance to antifolate drugs may affect the parasite’s ability to acquire essential nutrients or maintain cellular homeostasis, resulting in fitness costs in certain environments.^[34]^

#### 2.2.4. Influence on resistance spread

Parasites carrying drug resistance mutations may face a selective disadvantage in the absence of drug treatment due to the fitness costs associated with resistance. In settings where drug pressure is reduced or absent, susceptible parasites may outcompete resistant strains, leading to the suppression or elimination of resistant parasites within the population.^[35]^ Fitness costs associated with drug resistance mutations can influence transmission dynamics within parasite populations. Parasites with lower fitness may be less successful at establishing and maintaining infections in mosquito vectors or human hosts, resulting in reduced transmission rates and a decline in the prevalence of resistance over time.^[36–38]^

## 3. Molecular mechanisms of antimalarial drug resistance

Chloroquine resistance in Plasmodium falciparum is primarily associated with mutations in the pfcrt gene, particularly the K76T mutation. Other mutations in pfcrt, such as A220S, N326S, and I356T, may also contribute to chloroquine resistance.^[11,39]^ Mutations in the pfmdr1 gene, such as N86Y, Y184F, S1034C, N1042D, and D1246Y, have been implicated in modulating chloroquine resistance, although their roles may vary depending on parasite genetic background and drug pressure.^[22,40,41]^ Artemisinin resistance in *P. falciparum* has been linked to k13 propeller domain. Numerous mutations, including C580Y, R539T, Y493H, and I543T, have been associated with artemisinin resistance and delayed parasite clearance rates.^[12,42]^

While kelch13 mutations are the primary genetic determinants of artemisinin resistance, additional genetic loci may also contribute to the phenotype. These include mutations in genes involved in DNA repair (e.g., fd, arps10), lipid metabolism (e.g., ap2-g), and transcriptional regulation.^[21,43,44]^ Resistance to artemether–lumefantrine combination therapy can arise due to mutations in genes associated with drug met35olism, such as cytochrome P450 enzymes. Additionally, mutations in transporter proteins, such as pfmdr1, may also contribute to reduced drug susceptibility.^[41,45,46]^

Resistance to piperaquine, often used in combination therapies, can be attributed to mutations in genes involved in drug transport and metabolism, such as the plasmepsin II/III genes and the pfcrt. Amplification of the plasmepsin II/III genes has also been associated with piperaquine resistance.^[44,47,48]^ Similar to artemisinin resistance, resistance to artesunate, a derivative of artemisinin, has been linked to mutations in the kelch13 gene. These mutations impair the parasite’s susceptibility to artemisinin derivatives and may contribute to treatment failure.^[2,49]^

## 4. Population genetics methodologies for studying antimalarial drug resistance

### 4.1. Whole-genome sequencing (WGS)

WGS involves sequencing the entire genome of Plasmodium parasites, providing comprehensive information on genetic variation, including single nucleotide polymorphisms, insertions, deletions, and structural variants. This technique allows researchers to identify mutations associated with antimalarial drug resistance and study their distribution within parasite populations.^[43,50]^

### 4.2. Allele frequency analysis

Allele frequency analysis involves quantifying the frequency of specific genetic variants, such as drug resistance mutations, within parasite populations. This approach allows researchers to assess the prevalence and distribution of resistance alleles over time and across different geographic regions, providing insights into the spread and dynamics of drug resistance.^[51,52]^

### 4.3. Selective whole genome amplification (sWGA)

sWGA is a method used to enrich parasite DNA from low-parasitemia samples, such as dried blood spots, for subsequent whole-genome sequencing. By selectively amplifying parasite DNA, sWGA enables the efficient and cost-effective sequencing of Plasmodium genomes from limited starting material, facilitating population-level studies of genetic variation and drug resistance.^[50,53]^

### 4.4. Genome-wide association studies (GWAS)

GWAS involve scanning the entire genome of parasite populations to identify genetic variants associated with drug resistance phenotypes. By correlating genetic variation with drug response data, GWAS can pinpoint loci linked to resistance and provide insights into the genetic basis of drug resistance traits.^[9,52]^

### 4.5. Influence of factors on selection of resistant genotypes

Drug usage patterns, including the type of antimalarial drugs used, treatment regimens, and adherence to treatment protocols, can exert selective pressure on parasite populations, favoring the emergence and spread of resistant genotypes. Overuse or inappropriate use of antimalarial drugs can accelerate the selection of drug-resistant parasites by providing them with a survival advantage over susceptible strains.^[54,55]^

Host immunity plays a crucial role in shaping the dynamics of antimalarial drug resistance. Immune-mediated clearance of drug-sensitive parasites can create a selective environment favoring the survival and proliferation of drug-resistant strains. Conversely, acquired immunity to specific drug-resistant parasites may reduce their fitness advantage, influencing the prevalence of resistance in endemic settings.^[56,57]^

Transmission dynamics, including vector abundance, vectorial capacity, and human mobility, can impact the spread of resistant genotypes within parasite populations. High transmission settings facilitate the transmission of drug-resistant parasites, increasing the likelihood of their establishment and dissemination. Conversely, interventions targeting transmission, such as vector control measures, may help mitigate the spread of resistance.^[58,59]^

### 4.6. Spatial and temporal variation in antimalarial drug resistance

Genetic variation in antimalarial drug resistance genes can vary spatially and temporally due to factors such as population structure, gene flow, and selection pressures. Parasite populations in different geographic regions may exhibit distinct resistance profiles, reflecting local patterns of drug usage, transmission dynamics, and host immunity.^[51,60]^ The prevalence of antimalarial drug resistance can vary spatially and temporally in response to changes in drug policy, migration patterns, and transmission intensity. Areas with high levels of migration or frequent travel may experience the importation of resistant parasites, leading to localized outbreaks of drug resistance. Moreover, changes in drug policies, such as the introduction of new antimalarial drugs or treatment regimens, can influence resistance prevalence over time.^[43,49]^

Local transmission intensity, determined by factors such as vector abundance, vectorial capacity, and human behavior, can shape the spatial and temporal distribution of antimalarial drug resistance. Areas with high transmission intensity may experience intense selection pressure for drug resistance due to frequent exposure to antimalarial drugs, leading to higher resistance prevalence compared to areas with lower transmission intensity.^[55,61]^

### 4.7. Spatial and temporal dynamics of antimalarial drug resistance

Genetic variation in antimalarial drug resistance genes exhibits spatial and temporal variation influenced by factors such as parasite population structure, gene flow, and selective pressures. For instance, studies have shown distinct genetic profiles of drug resistance genes across different regions, reflecting local patterns of drug usage and transmission intensity.^[2,51]^ The prevalence of antimalarial drug resistance varies spatially and temporally due to dynamic factors like migration, changes in drug policies, and local transmission intensity. Areas experiencing high levels of human migration may import drug-resistant parasites, leading to localized outbreaks. Moreover, changes in drug policies, such as the introduction of new treatment regimens, can influence resistance prevalence over time.^[6,61]^

Human migration plays a significant role in the spatial spread of antimalarial drug resistance. Movement of infected individuals from regions with high resistance prevalence to areas with lower resistance levels can introduce resistant parasites into new environments, contributing to the expansion and dissemination of drug resistance. Conversely, migration of individuals from areas with low resistance prevalence may introduce susceptible parasites, influencing local resistance dynamics.^[62,63]^ Local transmission intensity, determined by factors such as vector abundance, vectorial capacity, and human behavior, influences the spatial and temporal patterns of antimalarial drug resistance. Regions with high transmission intensity may experience greater selection pressure for drug resistance due to frequent exposure to antimalarial drugs, leading to higher resistance prevalence compared to areas with lower transmission intensity.^[62]^

## 5. Evolutionary rationale for combination therapies

Combination therapies involve the simultaneous administration of multiple drugs with different mechanisms of action. By targeting multiple pathways essential for parasite survival, combination therapies reduce the likelihood of parasites developing resistance to all components simultaneously. This approach lowers the selection pressure for resistant genotypes, delaying the emergence and spread of drug resistance.^[64,65]^

Combination therapies can exhibit synergistic effects, where the combined action of individual drugs enhances their overall efficacy against malaria parasites. Synergy can result in more rapid parasite clearance and lower treatment failure rates compared to monotherapy, reducing the opportunity for resistant parasites to survive and proliferate.^[65,66]^

The use of combination therapies can delay the onset of resistance by requiring parasites to acquire multiple mutations simultaneously to confer resistance. Given the low probability of multiple mutations arising within the same parasite simultaneously, combination therapies effectively raise the genetic barrier to resistance, prolonging the useful therapeutic lifespan of antimalarial drugs.^[64,66]^

Combination therapies can prevent cross-resistance between individual drugs by targeting different biochemical pathways or cellular targets. If parasites develop resistance to one drug in the combination, the other drug(s) remain effective against the resistant parasites, ensuring continued therapeutic efficacy and reducing the risk of treatment failure.^[65,66]^

### 5.1. Drug cycling and rotation strategies

Drug cycling involves the periodic alternation of different antimalarial drugs or drug combinations over specified time intervals. The rationale behind drug cycling is to selectively apply different drug pressures to malaria parasite populations, thereby preventing the continuous selection of resistant genotypes to any single drug. By periodically withdrawing the use of a particular drug, cycling aims to reduce the prevalence of resistance and extend the useful therapeutic lifespan of antimalarial drugs.^[27,67]^

Drug rotation involves the sequential use of different antimalarial drugs or drug combinations in a predefined order. Unlike drug cycling, which involves periodic changes in drug usage patterns, drug rotation follows a predetermined sequence of drug deployment. The goal of drug rotation is to limit the duration of exposure to any single drug, thereby reducing the selection pressure for resistance and delaying the emergence of resistant genotypes.^[27,67]^

Both drug cycling and rotation aim to mitigate the evolution of antimalarial drug resistance by altering drug usage patterns. By periodically changing the drugs used for treatment, these strategies aim to disrupt the continuous selection pressure for resistant genotypes, reducing the opportunity for resistant parasites to proliferate and spread within parasite populations. Additionally, these approaches may also allow time for the reemergence of drug-sensitive parasites, restoring the effectiveness of previously used drugs.^[27,67]^

### 5.2. Influence of pharmacokinetic properties on antimalarial drug resistance

The pharmacokinetic properties of antimalarial drugs, including half-life and drug exposure, influence the selection pressures acting on malaria parasite populations. Drugs with longer half-lives and extended periods of drug exposure may exert greater selective pressure for resistance, as parasites are exposed to subtherapeutic drug concentrations for prolonged durations, providing opportunities for the emergence and proliferation of resistant genotypes.^[68,69]^

The rate of drug clearance from the body can impact the efficacy of antimalarial treatment and the development of resistance. Drugs with rapid clearance rates may require more frequent dosing, increasing the likelihood of suboptimal drug concentrations and promoting the selection of resistant parasites. Conversely, drugs with slower clearance rates may maintain therapeutic concentrations for longer durations, reducing the risk of resistance emergence.^[45,70]^

Variability in drug metabolism and distribution can influence the effectiveness of antimalarial treatment and the emergence of resistance. Differences in metabolism rates among individuals may result in variable drug exposure levels, affecting treatment outcomes and the selection of resistant parasites. Additionally, drugs that exhibit poor tissue distribution may fail to reach parasite reservoirs effectively, allowing parasites to persist and develop resistance.^[68,69]^

Pharmacokinetic interactions between antimalarial drugs and host factors, such as drug metabolism enzymes and transport proteins, can impact drug efficacy and resistance dynamics. Genetic polymorphisms in host enzymes involved in drug metabolism may affect drug clearance rates, altering drug exposure levels and influencing the selection of resistant parasites. Moreover, host immune responses and physiological factors can also influence drug distribution and effectiveness, impacting resistance evolution.^[45,70]^

### 5.3. Importance of genomic surveillance for monitoring antimalarial drug resistance

Genomic surveillance allows for the early detection of mutations associated with antimalarial drug resistance, providing crucial insights into the emergence and spread of resistant parasites. By monitoring genetic variations in parasite populations over time, genomic surveillance can identify novel resistance mutations before they become widespread, enabling proactive intervention strategies.^[47,71]^ Genomic surveillance facilitates the tracking of resistance spread across different regions and populations in real-time. By analyzing genetic data from diverse geographical locations, researchers can identify patterns of resistance transmission and assess the effectiveness of control measures. This information is essential for guiding targeted interventions and adapting treatment strategies to local resistance profiles.^[9,72]^

Genomic surveillance enables the characterization of underlying resistance mechanisms, elucidating the genetic basis of drug resistance and informing the development of novel therapeutics. By identifying genetic markers associated with resistance phenotypes, researchers can design molecular assays for rapid resistance detection and guide the selection of effective treatment regimens.^[47,71]^

Genomic surveillance plays a crucial role in monitoring for novel resistance threats and emerging resistance hotspots. By continuously monitoring genetic diversity in parasite populations, researchers can detect changes in resistance patterns and identify potential resistance hotspots before they become widespread. This proactive approach allows for timely interventions to prevent the spread of resistance and preserve the efficacy of existing antimalarial drugs.^[9,72]^

### 5.4. Adaptive management strategies for antimalarial drug resistance

Antimalarial drug resistance is a dynamic process shaped by evolutionary forces acting on parasite populations. The rapid evolution and spread of resistance necessitate adaptive management strategies that can respond to changing resistance dynamics in real-time. Static treatment approaches are inadequate in the face of evolving resistance, highlighting the need for adaptive strategies that account for evolutionary processes.^[47,73,74]^

Adaptive management strategies require continuous monitoring of resistance prevalence and genetic markers associated with resistance. By integrating genomic surveillance data with epidemiological information, healthcare authorities can identify emerging resistance hotspots and adjust treatment protocols accordingly. Regular surveillance enables the early detection of resistance and informs timely interventions to mitigate its spread.^[73,75,76]^

Adaptive management strategies advocate for flexibility in treatment policies to accommodate changing resistance profiles. This may involve implementing drug rotation or combination therapies based on local resistance patterns, rather than relying solely on standardized treatment regimens. By adapting treatment protocols to the evolving resistance landscape, healthcare systems can optimize therapeutic outcomes and prolong the effectiveness of available antimalarial drugs.^[47,74,75]^

Adaptive management strategies also involve community engagement and education to promote responsible antimalarial drug use and reduce the risk of resistance emergence. Educating healthcare providers and the general population about the importance of adhering to treatment protocols, avoiding counterfeit drugs, and adopting preventive measures such as vector control can help slow the spread of resistance and prolong the efficacy of antimalarial treatments.^[73,76,77]^

### 5.5. Emerging approaches for antimalarial drug development

Emerging approaches for antimalarial drug development aim to target novel pathways in the malaria parasite’s lifecycle, thereby minimizing the risk of resistance. By identifying essential biological processes that are not targeted by existing drugs, researchers can develop innovative therapeutics with distinct mechanisms of action. These novel drugs disrupt vital parasite functions, making it difficult for parasites to develop resistance through known mechanisms.^[78,79]^

Multi-targeted therapies represent another emerging approach for antimalarial drug development. Instead of targeting a single pathway, multi-targeted drugs simultaneously inhibit multiple essential processes in the parasite’s lifecycle. By disrupting multiple targets, these drugs impose a higher genetic barrier to resistance, as parasites would need to acquire mutations affecting multiple pathways to evade drug action effectively. Multi-targeted therapies have the potential to delay resistance emergence and prolong the efficacy of antimalarial treatment.^[78,79]^

Host-directed therapies represent an innovative approach to antimalarial drug development that targets host factors essential for parasite survival. By modulating host immune responses or cellular processes necessary for parasite invasion and replication, these therapies indirectly inhibit parasite growth and reduce the risk of resistance development. Host-directed therapies offer the advantage of targeting conserved host factors, potentially limiting the emergence of resistance and providing novel avenues for antimalarial treatment.^[78,80,81]^

## 6. Implications for treatment strategies

The identification of specific genetic mutations has practical implications for treatment. For example, detecting *kelch13* mutations can guide the use of ACTs. In regions where these mutations are prevalent, alternative treatments may be necessary to ensure efficacy. Moreover, understanding the fitness costs associated with resistance can inform the development of drug regimens that exploit these weaknesses, potentially slowing the spread of resistant strains.^[82]^

### 6.1. Public health policy considerations

Public health policies must adapt to the evolving landscape of antimalarial resistance. Continuous surveillance of genetic markers is essential for early detection of resistance patterns. The World Health Organization has emphasized the need for strategies to respond to antimalarial drug resistance in Africa, highlighting the importance of timely detection and response to emerging resistance.^[83,84]^

## 7. Practical implications for treatment strategies and public health policies

Recognizing the evolutionary mechanisms underlying drug resistance in malaria is crucial for informing effective treatment strategies and public health policies. Below is an in-depth exploration of practical approaches to address this challenge:

### 7.1. Surveillance and monitoring

Implementing robust surveillance systems to promptly detect resistance patterns is essential. The World Health Organization emphasizes strengthening surveillance to ensure timely responses to emerging resistance.^[84,85]^

### 7.2. Optimized drug use

Rationalizing the use of antimalarial drugs can reduce selective pressure. This includes adhering to treatment guidelines, avoiding monotherapies, and ensuring complete treatment courses to minimize the survival of partially resistant parasites. For instance, the National Malaria Control Program in Uganda advocates for correct malaria prevention and management measures, emphasizing adherence to treatment protocols.^[41,86,87]^

### 7.3. Combination therapies

Utilizing ACTs remains a cornerstone in malaria treatment. Combining drugs with different mechanisms of action reduces the likelihood of the parasite developing resistance to multiple agents simultaneously. However, recent studies have raised concerns about emerging resistance to artemisinin in Africa, underscoring the need for ongoing monitoring and adaptation of treatment strategies.^[88,89]^

### 7.4. Research and development

Investing in the development of new antimalarial compounds and vaccines is vital. Recent advancements, such as the RTS,S and R21 vaccines, offer promising avenues for reducing malaria incidence and, consequently, the reliance on drug treatments. The R21 vaccine, developed by Oxford University and the Serum Institute of India, has been introduced in several African countries, marking a significant step toward malaria eradication.^[90,91]^

### 7.5. Public health interventions

Integrating resistance management into broader malaria control programs, including vector control measures and public education campaigns, can mitigate the spread of resistant strains. For example, Brazil and Thailand have launched new single-dose radical cure medicines to prevent the relapse of Plasmodium vivax malaria, demonstrating the importance of comprehensive public health strategies.^[41,83,92,93]^

Evolutionary biology of antimalarial drug resistance, key findings, genetic basis, and implications for treatment and Public Health are summarized Table 1.

**Table 1:** Summary of evolutionary biology of antimalarial drug resistance, key findings, genetic basis, and implications for treatment & public health.

Aspect	Key findings	Genetic basis	Implications for treatment & public health	References
Mechanism of resistance	Resistance emerges due to genetic mutations under drug selection pressure.	*kelch13* (artemisinin resistance), *pfcrt* (chloroquine resistance), *pfmdr1* (multidrug resistance)	Targeted therapies and surveillance programs for early detection.	[41,44]
Spread of resistance	Resistance spreads through human migration, high transmission, and parasite reproductive dynamics.	High mutation rates in *P. falciparum* genes	GIS mapping, containment strategies, and drug policy modifications.	[37,38]
Fitness costs & evolutionary trade-offs	Resistant strains initially exhibit reduced fitness, but compensatory mutations restore viability.	Mutations in *kelch13* interact with other genes to balance fitness and resistance.	Exploiting fitness costs in drug design to limit resistant strain survival.	[31,32]
Host–parasite coevolution	Human immune responses and parasite adaptations drive resistance evolution.	Polymorphisms in *dhfr*, *dhps* genes (sulfadoxine-pyrimethamine resistance)	Personalized malaria treatment based on host genetic factors.	[81]
Epigenetic & non-genetic adaptations	Epigenetic changes (e.g., chromatin remodeling) enable temporary resistance without mutations.	Histone modifications linked to drug response	Novel drug targets addressing epigenetic mechanisms.	[74,76]
Impact on malaria control strategies	Resistance threatens elimination efforts, requiring adaptive drug policies and monitoring.	Molecular surveillance of resistance genes	Integrating genetic data into malaria control programs for effective interventions.	[41,83]

## 8. Conclusion

Antimalarial drug resistance is driven by dynamic evolutionary processes within parasite populations. These processes include natural selection acting on genetic variation, mutation, gene flow, and genetic drift. Resistance emerges and spreads in response to selective pressures exerted by antimalarial drugs, leading to the survival and proliferation of resistant parasite strains.^[1,2]^ Antimalarial drug resistance is mediated by specific genetic mutations in the parasite genome. These mutations can occur in genes encoding drug targets, transporters, or enzymes involved in drug metabolism. Different classes of antimalarial drugs target distinct biological pathways, and resistance mechanisms vary accordingly. Understanding the genetic basis of resistance is essential for developing effective treatment strategies and surveillance methods.^[3,4]^

Resistance mutations often incur fitness costs, reducing parasite fitness in the absence of drug pressure. However, compensatory evolution can mitigate these costs by restoring parasite fitness through secondary mutations or genetic mechanisms. Understanding the trade-offs between resistance and fitness is crucial for predicting the spread and persistence of resistant parasites in natural populations.^[5,6]^ Resistance prevalence and genetic variation within parasite populations exhibit spatial and temporal dynamics. Factors such as drug usage patterns, host immunity, migration, and transmission intensity influence the distribution and spread of resistance. Monitoring spatial and temporal trends in resistance prevalence is essential for guiding control efforts and optimizing treatment strategies.^[7,8]^

Evolutionary insights highlight the importance of dynamic treatment strategies that adapt to changing resistance dynamics. Antimalarial drug policies need to incorporate genomic surveillance data and evolutionary principles to optimize treatment guidelines. Flexibility in treatment protocols, such as drug rotation and combination therapies, can help mitigate resistance emergence and spread.^[1,2]^

Evolutionary insights emphasize the need for robust surveillance and monitoring systems to detect resistance emergence and track its spread. Genomic surveillance techniques enable the early detection of resistance mutations and provide valuable data for guiding treatment policies. Regular monitoring of resistance prevalence and genetic diversity within parasite populations is essential for informing control efforts and preserving treatment efficacy.^[3,4]^

Evolutionary insights underscore the importance of regional and global collaboration in tackling antimalarial drug resistance. Collaboration among affected countries, researchers, healthcare providers, and policymakers is essential for sharing data, coordinating surveillance efforts, and implementing effective control measures. By fostering collaboration and information exchange, the global community can enhance its capacity to respond to emerging resistance threats.^[5,6]^

Evolutionary insights drive research and innovation in antimalarial drug development. Understanding the genetic basis of resistance and the underlying evolutionary processes informs the design of new therapeutics with improved efficacy and resistance profiles. Innovations such as novel drug targets, multi-targeted therapies, and host-directed approaches offer promising avenues for overcoming resistance challenges and advancing malaria control efforts.^[7,8]^

## 9. Recommendation

Future research should focus on elucidating novel mechanisms of antimalarial drug resistance beyond those currently characterized. Investigating the genetic basis of resistance in diverse parasite populations and exploring unconventional pathways targeted by new drug candidates can uncover previously unknown resistance mechanisms. Understanding these mechanisms is crucial for developing effective treatments that minimize the risk of resistance emergence.

Investigating host–parasite interactions and their impact on resistance evolution can provide valuable insights into malaria pathogenesis and treatment outcomes. Future research should explore host genetic factors influencing susceptibility to infection and treatment response, as well as the role of host immunity in shaping parasite diversity. Understanding the complex interplay between host and parasite biology is essential for developing personalized treatment approaches and vaccines.

Additionally, research into combination therapies and drug synergy can optimize treatment regimens and delay the emergence of resistance.

## Author contributions

**Conceptualization:** Matthew Chibunna Igwe.

**Writing – original draft:** Matthew Chibunna Igwe, Ogbonna Alphonsus Ogbuabor.

**Writing – review & editing:** Matthew Chibunna Igwe, Ogbonna Alphonsus Ogbuabor, Emmanuel Ifeanyi Obeagu.
